# Huoxue Qianyang Qutan Recipe Protects against Early Renal Damage Induced by Obesity-Related Hypertension via the SIRT1/NF-*κ*B/IL-6 Pathway: Integrating Network Pharmacology and Experimental Validation-Based Strategy

**DOI:** 10.1155/2022/9599090

**Published:** 2022-05-27

**Authors:** Mingzhu Wang, Jianhua Li, Mingtai Gui, Bo Lu, Lei Yao, Xunjie Zhou, Moyi Shi, Liang Hu, Deyu Fu

**Affiliations:** ^1^Yueyang Hospital of Integrated Traditional Chinese and Western Medicine, Shanghai University of Traditional Chinese Medicine, Shanghai, China; ^2^Academy of Integrative Medicine, Shanghai University of Traditional Chinese Medicine, Shanghai, China

## Abstract

Obesity is recognized as not only a major contributing factor to cardiovascular diseases but also an independent risk factor for end-stage renal disease. Previous studies have found that Huoxue Qianyang Qutan Recipe (HQQR) could reduce urinary microalbumin in patients with obesity-related hypertension (OBH). However, the renal protective activity of HQQR in OBH and its molecular targets involved remains ambiguous. In this work, we investigate the mechanism of HQQR against OBH-induced early renal damage using integrating network pharmacology and experimental validation-based strategy. First, via network pharmacology, IL-6 is identified as one of the key targets of HQQR against early renal damage in hypertension, and inhibition of inflammation is a crucial process. Second, in in vivo experiments, HQQR can lower blood pressure, lose weight, and restore metabolic abnormalities in OBH rats, which could be associated with the effects on protecting early renal damage. Finally, in the mechanism, HQQR increases SIRT1 mRNA and protein expression consistent with reduction of NF-*κ*B acetylation and suppressed the p65-mediated inflammatory signaling pathway. As a result, HQQR robustly inhibits OBH-induced renal inflammation by reducing IL-6 mRNA and protein levels in the renal tissue and the release of IL-6 in serum of OBH rats. This study aims to provide a multimethod (network pharmacology-animal experiment) and multilevel (component-target-pathway) strategy for the prevention and treatment of OBH-induced target organ damage by traditional Chinese medicine.

## 1. Introduction

Hypertension is the leading risk factor for death worldwide [1]. Excess weight gain, as a major cause of hypertension, accounts for 65–75% of the hypertensive risk [2]. With prolonged obesity, obesity-related hypertension (OBH) contributes directly to cardiovascular disease (CVD) and target organ damage (TOD), especially renal injury [3]. OBH becomes more difficult to control due to dyslipidemia, insulin resistance, and inflammation, often requiring multiple antihypertensive drugs and treatment of other risk factors [4].

Major TOD of OBH includes higher prevalence of hypertension-associated cardiorenal and metabolic disorders. Nevertheless, the mechanisms of renal injury induced by TOD have not been fully elucidated. Accumulating evidences unravel that inflammation and the immune system which interact synergistically with OBH may cause renal injury [5, 6]. Meanwhile, many investigations have also focused on the close molecular coordination between the inflammation and energy metabolic supply in OBH [7, 8], suggesting that chronic inflammation with metabolic abnormalities accounts for a far higher proportion of renal damage and CVD [9]. Therefore, new multifunctional agents to reduce the risk of end-stage renal diseases induced by OBH face a major challenge owing to the pathogenic mechanisms attributed to multiroute and multitarget pathways.

Traditional Chinese medicine (TCM) as a complementary medicine is becoming increasingly available worldwide. Chinese herbs, as a representative of multitarget interventions, have been proved useful in relieving hypertension-related symptoms [10, 11]. It has recently been shown that Huoxue Qianyang Qutan Recipe (HQQR) could be effective in left ventricular hypertrophy and cardiac remodeling in OBH rats. The mechanism may be relevant to improving mitochondrial function through the SIRT1/PGC-1*α* deacetylation pathway and ATF6-CHOP endoplasmic reticulum stress signaling pathway [12, 13]. Meanwhile, we also found that HQQR can reduce the urinary microalbumin level in patients with OBH [14], suggesting that HQQR may protect against renal injury. However, the mechanism of HQQR against hypertensive renal damage has not been elucidated.

Network pharmacology as an interdisciplinary subject can predict potential gene targets and the molecular mechanism of drugs on diseases by analyzing the multilevel network of “diseases-genes-drug targets” [15]. It drives the modernization and mechanism research of TCM formulas [16]. Herein, we aim to explore the potential targets and pathways of HQQR against the early renal damage induced by OBH using integrating network pharmacology and experimental validation-based strategy.

## 2. Materials and Methods

### 2.1. Screening of Active Components and Related Targets

Traditional Chinese Medicine Systems Pharmacology Database and Analysis Platform (TCMSP) database [17] (http://tcmspw.com/tcmsp.php, Ver.2.3) and Bioinformatics Analysis Tool for Molecular mechANism of Traditional Chinese Medicine (BATMAN-TCM) database [18] (http://bionet.ncpsb.org/batman-tcm/, updated January 2016) were utilized to screen all compounds of HQQR. These compounds that met two requirements of oral bioavailability (OB) of ≥30% and drug likeness (DL) of ≥0.18 were further screened as bioactive components [17]. TCMSP and DrugBank (https://www.drugbank.ca/, version 5.1.5) databases were used to obtain the targets related to the HQQR bioactive components. The UniProt database (http://www.uniprot.org/) was applied to convert the overannotation protein names to standardized gene symbols [19].

### 2.2. Prediction of Disease Targets

The hypertensive renal damage-related targets were obtained via GeneCards [20] (https://www.genecards.org, version 4.1.4) and OMIM [20] (http://www.omim.org, updated March 25, 2020) databases. The compound targets and disease targets were intersected by the R software to obtain the therapeutic targets of HQQR against hypertensive renal damage.

### 2.3. Biological Functional Annotation

The therapeutic targets of HQQR were analyzed to explore the biological functional annotation (GO and KEGG) by “BiocManager” R package [21].

### 2.4. Network Analysis

The therapeutic targets were imported into STRING (https://string-db.org/, version 11.0) database [22] to get the PPI (protein-protein interaction) network using a high confidence score (correlation degree ≥0.900), as the cutoff value. Compound-target network construction was performed by Cytoscape 3.72 (https://cytoscape.org/). CytoHubba was employed to pick out hub nodes with high degrees of connectivity in the network by investigating the node composition.

### 2.5. OBH Rats and Drug Administration

120 male spontaneously hypertensive rats (SHR) and age/sex-matched Wistar–Kyoto rats (WKY) (five-week-old, 150 ± 20 g) were obtained from the Vital River Laboratory Animal Technology Co., Ltd. (animal license number: SCXK (Beijing) 2016–0006). The animal procedures were approved by the Institutional Animal Care and Use Committee at Yueyang Hospital in accordance with the principles outlined in the NIH guidelines for the care and use of laboratory animals (no. 18922).

Valsartan capsule (batch number: H20040217) was manufactured by Novartis Pharmaceutical Factory (Beijing, China).

HQQR, consisted of *Salvia miltiorrhiza*, stone cassia, *Ligusticum chuanxiong*, *Uncaria angustifolia*, corn whisker, mulberry parasite, and hawthorn (5 : 10 : 3:5 : 10 : 5:5), was decocted and dried following common protocol [12].

### 2.6. Experimental Procedure

The method of modeling obese rats was referred to early research [23]. The normal diet (no. P1101F) and high-fat diet were purchased from Shanghai Puluteng Biotechnology Co., Ltd. The rats were under a 12/12 h light/dark period cycle at controlled temperature (22 ± CA). The specific workflow followed is shown in Figure 1.

OBH model preparation: with WKY-normal diet and SHR-normal diet as control, SHR high-fat diet was evaluated to prepare OBH models, including 3 groups: WKY-normal diet (WKY-ND), SHR-normal diet (SHR-ND), and SHR high-fat diet (SHR-HF). After feeding a high-fat diet of 10 weeks, SHR-HF with weight in the upper third was selected as obese hypertensive rats (OBH rats).

Drug intervention: the rats were divided into four groups: WKY-normal diet (WKY), OBH high-fat diet (OBH), OBH high-fat diet and 30 mg/kg/d of valsartan by gavage (OBH-V), and OBH high-fat diet and HQQR (38.7 g/kg/d) by gavage (OBH-H).

### 2.7. Biochemical Detection

Whole blood was drawn from the abdominal aorta and centrifuged to isolate rat plasma samples. Then, mAlb (microalbuminuria), UCr (urine creatinine), NAG (urinary N-acetylglucosamine polyase), TC (total cholesterol), TG (triglyceride), LDL-C (low-density lipoprotein-cholesterol), HDL-C (high-density lipoprotein-cholesterol), and FPG (fasting plasma glucose) levels were detected by enzymatic kits (Nanjing Jiancheng Bioengineering Institute, Nanjing, China) using a digital UV spectrophotometer (mode SL-159, Elico Ltd., Telangana, India). The concentration of IL-6 (interleukin-6), Cys-C (Cystatin C), and FIN (fasting insulin) was determined with the help of radioimmunoassay kits (Beijing North Institute of Biological Technology, Beijing, China) according to the manufacturer's instructions. HOMA-IR (homeostasis model assessment of insulin resistance) = (FPG, mmol/L) × (FIN, *μ*IU/ml)/22.5.

### 2.8. Hematoxylin and Eosin (H&E) Staining and Transmission Electron Microscopy

The renal cortex tissues sections (5 *μ*m thick) were subjected to H&E staining. An optical microscope (Leica, Germany) was used to photograph and analysis at 400× magnification. Renal tissues (1 cubic millimeter) at renal cortex were separated and fixed in 2.5% glutaraldehyde for 2 h at 4°C, and the ultrastructure was observed under the transmission electron microscope (FEI Tecnai G2 Spirit, Thermo Fisher Scientific, U.S.A.) at 6000 × magnification.

### 2.9. RNA Extraction and Quantitative Real-Time PCR (qRT-PCR)

The renal cortex tissues were used to perform RNA extraction and qRT-PCR as previously described [24]. The relative mRNA level was obtained by calculating 2^−ΔΔ*C*_*T*_^. GAPDH (glyceraldehyde-3-phosphate dehydrogenase) was the inner control for normalization. The primer sequences were presented as follows: 5′-GGTTAGGTGGCGAGTATGC-3 and 5′-TATGAAGAGGTGTTGGTGGC-3′ for SIRT1 (silent information regulator 1); 5′-CAGCCACTGCCTTCCCTAC-3′ and 5′-CAGAATTGCCATTGCACAAC-3′ for IL-6; and 5′-GGAGTCTACTGGCGTCTTCAC-3′ and 5′-ATGAGCCCTTCCACGATGC-3′ for GAPDH.

### 2.10. Western Blotting

The total proteins extracted from renal cortex tissues were separated by SDS-PAGE and were transferred to the PVDF membrane. After blocking in 5% nonfat milk for 1 h, protein bands were incubated with primary antibodies, followed by incubation with corresponding second antibodies. Protein bands were visually measured by a chemiluminescent imaging system (Tanon, Shanghai, China). Anti-SIRT1 (Ab110304, 1 : 1000), anti-NF-*κ*B/*p*65 (Ab16502, 1 : 2000), and anti-IL-6 (Ab233706, 1 : 1000) antibodies were purchased from Abcam. Anti-GAPDH (60004-1-1G, 1 : 5000) antibody was purchased from Proteintech, and anti-ac-p65 (Bs-23216R, 1 : 500) antibody was provided by Bioss.

### 2.11. Data Analysis

All data were plotted using GraphPad Prism 8.0 (San Diego, CA, USA). Data were expressed as mean ± standard error of the mean (SEM). The normality test was performed via the Shapiro–Wilk test. The statistical software SPSS 26.0 (SPSS Ltd., U.S.A.) was used for statistical analysis. Analysis of variance (ANOVA) with Turkey's posthoc test was used for comparison between the means of multiple groups. A *P* value ≤0.05 was considered statistically significant.

## 3. Results

### 3.1. IL-6 Is Identified as the Key Target of HQQR against Hypertensive Renal Damage

Totally, 4320 targets of hypertensive renal damage were screened using GeneCards and OMIM databases. 167 targets of the ingredients in HQQR were obtained from the TCMSP database. Among these 167 HQQR-related targets, 158 genes were closely related to hypertensive renal damage (Figure 2(a)). Then, 158 therapeutic targets were input to the STING database to get the PPI network. Top 20 hub genes were screened out using CytoHubba in the Cytoscape software. Among these 20 top genes, cytokines (IL-6, IL-10, IL-4, and IL-1*β*) take a higher proportion, especially IL-6 (Figure 2(b)). Therefore, IL-6 was identified as the key target of HQQR against hypertensive renal damage and further studied in later animal experiments.

Through the TCMSP database, 598 compounds were retrieved from HQQR. Then, we selected OB ≥ 30% and DL ≥ 0.18 as the bioactive components to get 118 bioactive herbal compounds. Moreover, we further constructed an interaction network between top 20 hub gene targets (green arrow) and herbal compounds. Through network analysis, 35 core herbal compounds (blue circle) were obtained, including isocorynantheic acid, quercetin, coryincine, stigmast-7-en-3-ol, mandenol, chryseriol, stigmasterol, luteolin, schottenol, hirsutaside C, hirsutine, yohimbine, hirsutaside B, corynoxeine, sitosterol, and kaempferol (Figure 2(c)). Interestingly, *Salvia miltiorrhiza* (Danshen), which is also the principal drug (Junyao or monarch drug) of HQQR, is identified as the main component.

### 3.2. Evaluation of the Obesity-Related Hypertension Rat Model

36 (top 1/3) obesity rats were selected as OBH rat models. From Figures 3(a) and 3(b), we can find that the body shape of OBH rats was significantly larger than that of the SHR-normal diet (SHR-ND). Meanwhile, the content of perirenal fat increased evidently. Compared with SHR-ND, the systolic blood pressure (SBP), weight, and waist circumference of the OBH group were significantly increased (*p* < 0.001) (Figures 3(c), 3(d) and 3(e)).

### 3.3. HQQR Controls Blood Pressure, Weight, and Abdominal Circumference in OBH Rats

Compared with the OBH model group, the weight and abdominal circumference were significantly decreased after 8 weeks (*p* < 0.05). Moreover, the body weight and abdominal circumference in the HQQR group are evidently lower than that of the valsartan group (*p* < 0.05). HQQR could obviously control both SBP and DBP after treatment for 2 weeks (*p* < 0.05). The antihypertensive effect of HQQR equals that of valsartan after 6 weeks of intervention. HQQR can control blood pressure more smoothly than valsartan (Figures 3(f)–3(i)).

### 3.4. HQQR Protects against Early Renal Damage in OBH Rats

Many studies have investigated the association between renal tubular damage markers (mAlb, UCR, NAG, and Cys-C) and the development and progression of early stage renal damage because of their clinical relevance which are sensitive and specific for predicting renal glomerulopathy [25–27]. Our results show that HQQR can decrease mAlb, UCR, NAG, and Cys-C, compared with OBH groups (*p* < 0.05 or *p* < 0.01) (Figure 4(a)). In addition, the level of serum IL-6 was markedly reduced after HQQR treatment (*p* < 0.01) (Figure 4(b)).

We further observed the pathological changes of glomeruli by H and E staining. The results exhibit that many inflammatory cells were infiltrated around the glomerulus or accompanied by renal tubular atrophy or disappearance in OBH groups. HQQR reduces the accumulation of inflammatory cells and recover the glomerular normal structure (Figure 4(c)).

The changes of the renal structure may not be obvious in the early stage. Therefore, the ultrastructure of renal cortex tissues was further observed under the transmission electron microscope. We discover podocyte fusion or degeneration, even endothelial cell apoptosis, local thickening of mesangial area, and thinning of mesangial interstitium in OBH groups. However, the abovementioned changes were alleviated in the HQQR group (Figure 4(d)).

### 3.5. HQQR Improves Metabolic Abnormalities in OBH Rats

Apparently, OBH is always accompanied by metabolic abnormalities. Consequently, the evaluation of metabolic-related indicators is of vital importance. Compared with the OBH group, HQQR reduces the levels of FPG and HOMA-IR (*p* < 0.01 or *p* < 0.05) (Figures 5(a) and 5(b)). Meanwhile, the levels of TC, TG, and LDL-C are also decreased, and HDL-C is increased in the HQQR group (*p* < 0.05 or *p* < 0.01) (Figures 5(c)–5(f)). These results suggest that HQQR can regulate the metabolism, which is one of the potential mechanisms of protecting against OBH-induced early renal damage.

### 3.6. HQQR Upregulated SIRT1 Expression in the Renal Tissue of OBH Rats

SIRT1 can deacetylate histones and nonhistone proteins to regulate the cell metabolism throughout the body. Our results demonstrated that both mRNA and protein levels of SIRT1 are evidently decreased in the OBH group, compared with the WKY group. HQQR treatment completely prevents the downregulation of SIRT1 mRNA and protein expression (*p* < 0.001) (Figures 6(a), 6(b) and 6(c)).

### 3.7. HQQR Reduced NF-*κ*B Acetylation (Ac-NF-*κ*B) and Suppressed the p65-Mediated Inflammatory Signaling Pathway in the Renal Tissue of OBH Rats

NF-*κ*B signaling plays a major role in innate immunity defense; meanwhile, NF-*κ*B p65 is a substrate of SIRT1. Compared with WKY groups, the acetylation of p65 markedly increased in the renal tissue of OBH rats, and this upregulation was suppressed by HQQR (*p* < 0.05) (Figures 6(a)–6(c) and 6(d)). Concurrently, HQQR completely suppressed OBH-induced p65 nuclear translocation in the renal tissue. As a result, HQQR robustly inhibited OBH-induced neuroinflammation by reducing IL-6 mRNA and protein levels (*p* < 0.05 or *p* < 0.01) (Figures 6(a)–6(f)).

## 4. Discussion

In the present work, we proposed an integrated strategy via network analysis and experimental validation to illustrate the mechanisms of HQQR against early renal damage induced by OBH systematically. First, previous works of our team have demonstrated that HQQR regulated mitochondrial function and protected hypertensive myocardial hypertrophy through upregulating the expression of SIRT1. Second, via network pharmacology, IL-6 is identified as a key target of HQQR against hypertensive kidney damage; in addition, inflammation is one of the hub pathological processes. Third, recent studies have indicated that the interrelation of inflammation and energy metabolism leads to target organ damage of obesity and hypertension. Consequently, SIRT1/NF-*κ*B/IL-6, which represents the classic signaling pathways to regulate metabolic and inflammatory networks, was one of the potential mechanisms of OBH renal damage.

Obesity, due to its strong association with diabetes and hypertension, is considered as the crucial risk factor for chronic and end-stage kidney diseases [28]. OBH accompanied by the higher energy metabolism, which is caused by the interaction of adipose and IR (insulin resistance), provides “soil” for the chronic inflammation-induced TOD. The inflammatory process and metabolic abnormalities cause the initiation and progression of OBH-induced renal damage [29]. Our results indicated that HQQR is proven to be stable and effective in treating hypertension. Concurrently, HQQR also improved metabolic abnormalities in OBH rats including reducing serum FBG and HOMA-IR levels, consistent with decreased serum TG, TC, and LDL-C levels and increased HDL-C levels. It has been confirmed that IR is the common pathological mechanism of hypertension combined with metabolic-related diseases (such as abdominal obesity, glucose and lipid metabolism disorder, uric acid abnormality, and so on) [30, 31]. Therefore, the improving insulin resistance effect of HQQR is crucial for the protection of TOD induced by OBH.

Protein acetylation has been identified as a novel therapeutic strategy to prevent the development and progression of CVDs including hypertension, cardiac hypertrophy, and heart failure [32]. Sirtuins are classiﬁed as deacetylases, especially SIRT1, which has been extensively studied [33]. In the kidneys, SIRT1 deacetylates target proteins to inhibit renal inflammation and fibrosis via multiple signal pathways [34]. Accumulating evidence has demonstrated that SIRT1 regulates blood pressure, glucose-lipid metabolism, and sodium balance [35–37], which also played an important role in kidney diseases. Accordingly, the activation of SIRT1 in the kidney may be a new therapeutic target to rectify independent risk factors of renal diseases, especially OBH renal damage.

The NF-*κ*B signal pathway plays a pivotal part in many inflammatory factors' expression [38]. In our work, we found that the mRNA and protein expression of SIRT1 is evidently decreased and that of Ac-NF-*κ*B p65 and inflammation-related IL-6 mRNA and protein expression levels significantly increased in the kidneys of OBH rats, compared with WKY rats. The increased levels of IL-6 both in the kidney and serum of OBH rats were reversed by HQQR, as well as of acetylated NF-*κ*B and consistent with the restoration of SIRT1 gene and protein expression in the kidney. Consequently, the increased levels of Ac-NF-*κ*B p65 owing to decreased SIRT1 protein expression can lead to OBH renal inflammation, whereas HQQR exhibits anti-inflammatory effects and renal protective activity by restoring SIRT1 expression in the kidney of OBH rats. Therefore, the in-depth study of immunity and inflammation will provide potential intervention targets for the prevention and treatment of TOD in hypertension.

Recent research suggests that IL-6 secretion caused by anxiety and stress, which can lead to the changes in the fatty inflammation microenvironment, is a main mechanism of obesity. IL-6 is secreted in brown adipocytes, causing brown adipocytes to fail to regulate the metabolism of glucose and to decompose fat, which ultimately leads to obesity [39]. Studies have reported that chemokines (such as TNF-*α* and IL-6) are involved in the formation of hypertension [40]. Compared with normal people, the levels of serum IL-1*β* and IL-18 are higher in patients with hypertension [41]. The application of anti-inflammatory therapy in hypertension is increasing. A new anti-inflammatory drug VA694 can slow down the development of hypertension [42]. Combined with our study, we find that many inflammatory cells infiltrate around the glomerulus of OBH rats, and HQQR treatments reduce inflammation. The above results provide strong theoretical support for our study, in which IL-6 was a core target of OBH renal damage identified by network pharmacology. Confidently, the studies of hypertension and its TOD from the perspective of inflammation will be more and more extensive and profound in the future works.

## 5. Conclusion

In the present work, integrating network pharmacology and experimental validation-based strategy were used to explore the potential mechanism of HQQR against OBH renal damage. HQQR can increase the expression of SIRT1 consistent with reduction of the NF-*κ*B acetylation expression level. Furthermore, HQQR reduces the mRNA and protein expression level of IL-6 in tissue and release of IL-6 in serum. These findings indicate that upregulating or activating SIRT1 and then reducing inflammation may be a promising therapeutic strategy for OBH-induced renal damage, and clinical trials of HQQR renal protective activity are warranted.

## Figures and Tables

**Figure 1:** Workflow for HQQR intervention in OBH-induced early renal damage.

**Figure 2:** (a) The therapeutic targets of HQQR against early renal damage. (b) The hub gene network of HQQR against early renal damage. (c) The hub target and core compound network of HQQR against early renal damage.

**Figure 3:** (a) Comparison of rat body size: the left is SHR-normal diet and the right is SHR-high-fat diet (OBH). (b) Comparison of rat perirenal fat: the left is SHR-normal diet and the right is SHR high-fat diet (OBH). (c) Comparison of SBP after the OBH model established. (d) Comparison of weight after the OBH model established. (e) Comparison of abdominal circumference after the OBH model established. (f) Comparison of SBP after drug treatment. (g) Comparison of DBP after drug treatment. (h) Comparison of weight after drug treatment. (i) Comparison of abdominal circumference after drug treatment. ^*∗∗∗*^*P* < 0.001.

**Figure 4:** (a) Comparison of mAlb, UCr, NAG, and Cys-C after drug treatment. (b) Comparison of IL-6 in serum after drug treatment. (c) Comparison of renal tissue H&E staining after drug treatment (400^*∗*^ magnification). (d) Comparison of renal tissue ultrastructure after drug treatment. ^*∗*^*P* < 0.05; ^*∗∗*^*P* < 0.01; ^*∗∗∗*^*P* < 0.001; ^*∗∗∗∗*^*P* < 0.0001.

**Figure 5:** (a) Comparison of FPG in serum after drug treatment. (b) Comparison of HOMA-IR in serum after drug treatment. (c) Comparison of TG in serum after drug treatment. (d) Comparison of TC in serum after drug treatment. (e) Comparison of LDL-C in serum after drug treatment. (f) Comparison of HDL-C in serum after drug treatment. ^*∗*^*P* < 0.05; ^*∗∗*^*P* < 0.01; ^*∗∗∗*^*P* < 0.001; ^*∗∗∗∗*^*P* < 0.0001.

**Figure 6:** (a) The protein expression of SIRT1, Ac-NF-*κ*B, NF-*κ*B, and IL-6 determined by immunoblotting. (b) Comparison of SIRT1 protein expression after drug treatment. (c) Comparison of SIRT1 mRNA expression after drug treatment. (d) Comparison of Ac-NF-*κ*B protein expression after drug treatment. (e) Comparison of IL-6 protein expression after drug treatment. (f) Comparison of IL-6 mRNA expression after drug treatment. ^*∗*^*P* < 0.05; ^*∗∗*^*P* < 0.01; ^*∗∗∗*^*P* < 0.001; ^*∗∗∗∗*^*P* < 0.0001.

## Data Availability

The data used to support the findings of this study are available from the corresponding author upon request.
